The article "MDST-DGCN: A Multilevel Dynamic Spatiotemporal Directed Graph Convolutional Network for Pedestrian Trajectory Prediction" was published in 2022. Journal: Comput Intell Neurosci.

# MDST-DGCN: A Multilevel Dynamic Spatiotemporal Directed Graph Convolutional Network for Pedestrian Trajectory Prediction

**DOI:** 10.1155/2022/4192367

**Published:** 2022-04-12

**Authors:** Shaohua Liu, Haibo Liu, Yisu Wang, Jingkai Sun, Tianlu Mao

**Affiliations:** ^1^School of Electronic Engineering, Beijing University of Posts and Telecommunications, Beijing 100876, China; ^2^Beijing Key Laboratory of Mobile Computing and Pervasive Device, Institute of Computing Technology, Chinese Academy of Sciences, Beijing 100190, China

## Abstract

Pedestrian trajectory prediction is an essential but challenging task. Social interactions between pedestrians have an immense impact on trajectories. A better way to model social interactions generally achieves a more accurate trajectory prediction. To comprehensively model the interactions between pedestrians, we propose a multilevel dynamic spatiotemporal digraph convolutional network (MDST-DGCN). It consists of three parts: a motion encoder to capture the pedestrians' specific motion features, a multilevel dynamic spatiotemporal directed graph encoder (MDST-DGEN) to capture the social interaction features of multiple levels and adaptively fuse them, and a motion decoder to produce the future trajectories. Experimental results on public datasets demonstrate that our model achieves state-of-the-art results in both long-term and short-term predictions for both high-density and low-density crowds.

## 1. Introduction

The task of pedestrian trajectory prediction is to predict pedestrians' future trajectories given their historical trajectories in the scenario. Pedestrian trajectory prediction plays a notable role in many aspects, such as automatic driving [1] and robot navigation [2–5]. To predict an accurate trajectory, only considering the historical trajectory of the target pedestrian is not enough. Other pedestrians' influences on the target pedestrian, which are called “social interaction features,” can often help make a better prediction. With the longer prediction horizon and denser crowds, the temporal correlations in the trajectories between current and previous time steps grow weaker and the impact of interactions on pedestrians' motion grows stronger.

To model social interactions, traditional methods use rule-based functions [6–10]. While rule-based methods can only capture simple interactions, data-driven methods use neural networks to automatically extract the social interaction features from the data, which can make use of the interaction features more effectively. Many data-driven methods obtained social interaction features based on pooling [11–14] or attention mechanisms [1, 15–20]. The graph convolutional neural networks have developed rapidly in recent years, and the graph structure is naturally suitable for directly describing the interactions between pedestrians. As a result, graph convolutional neural networks [21–25] have achieved excellent results in pedestrian trajectory prediction.

The article "MDST-DGCN: A Multilevel Dynamic Spatiotemporal Directed Graph Convolutional Network for Pedestrian Trajectory Prediction" was published in 2022. Journal: Comput Intell Neurosci.

Although there are many graph convolutional neural network-based methods, they do not make full use of them. For example, Social-BiGAT [21] only uses the graph representation as the pooling mechanism on the states of the recurrent neural networks. The new methods STGAT [22] and Social-STGCNN [23] constructed spatiotemporal graphs to model social interactions and achieved excellent results in predictions.

However, they ignore a crucial point that even if the social interactions with nearby pedestrians or distant pedestrians are of the same type, they will result in different actions of the target pedestrian. As shown in Figure 1, at time steps *t*_1_ and *t*_2_, when the target pedestrian marked with the red circle avoids the nearby pedestrians and the distant pedestrians, respectively, his avoidance movements will be different. The former is a sudden avoidance producing a trajectory with high curvature, while the latter is an early avoidance producing a trajectory with low curvature. Moreover, with the increase in prediction horizon, pedestrians far from the target pedestrian may become more important. From time step *t*_1_ to *t*_2_, pedestrian B has little impact on the target pedestrian, but in the total period from *t*_1_ to *t*_3_, the merging of them is the main factor affecting the target pedestrian's trajectory. In other words, the influence of nearby pedestrians is mainly sudden and short-term, while faraway pedestrians have long-term effects on the target pedestrian's movement tendency.

Most previous methods [21–25] use a single graph to model these two types of influences and tend to capture “average social interaction features.” However, these two types of influences are more suitable to be modeled separately at different levels of a multilevel graph. Besides, many methods [23, 25] build an undirected graph to model social interactions. However, social interactions between pedestrians are nonsymmetrical. Therefore, building a digraph is more suitable for social interactions. Other methods [24] build a directed graph by predefined rules, such as inserting edges from all people inside the view area. But predefined rules are incomplete. For example, a pedestrian may slow down to wait for his companion without looking at him. Thus, a data-driven way to build a directed edge is much better.

To address the limitations of these works, we propose a multilevel dynamic spatiotemporal directed graph representation to model the interactions between pedestrians comprehensively. In our graph, different levels model interactions of pedestrians at different distance ranges. As shown in Figure 1, whether there is a spatial edge from a pedestrian to the target pedestrian at a level depends on whether their distance is within the corresponding distance range. With the change of time, the spatial edge between two pedestrians may break at one level and link at another. Even if the edge keeps linking at the same level, the influence of the neighbour also changes dynamically over time. To process the multilevel graph, we propose a multilevel dynamic spatiotemporal digraph convolutional network (MDST-DGCN). At each level of the graph, we use a node aggregator architecture to generate social interaction embedding by sampling and aggregating features from a node's spatial neighborhood like GraphSAGE [26]. Because social interactions are location independent, we do an aligning operation before aggregating features, which can advance performance significantly. Through the orderly use of sampling, aligning, and aggregating, the aggregator architecture becomes a naturally data-driven way to describe a directed edge. For each level of the graph, after the spatial interactions are captured, an LSTM [27] is used to capture the temporal correlations of interactions. And then, MDST-DGCN fuses interaction features of all levels adaptively. Through modelling social interactions at different levels, our multilevel dynamic spatiotemporal digraph convolutional network (MDST-DGCN) can fully extract pedestrians' social interaction features.

The article "MDST-DGCN: A Multilevel Dynamic Spatiotemporal Directed Graph Convolutional Network for Pedestrian Trajectory Prediction" was published in 2022. Journal: Comput Intell Neurosci.

In summary, our contribution is twofold. First, we propose using the spatiotemporal dynamic map with a multilevel concept to separate pedestrian nodes, resulting in varying effects on the trajectory depending on the distance between pedestrians, which may aid in the extraction of social interaction features by partitioning pedestrian distances at various levels. Second, we create an aggregator based on the GraphSAGE that converts the original static adjacency graph structure into a dynamic directed graph structure by sampling, aligning, and aggregating, reducing the effect of individual coordinates on the model and the overfitting phenomenon. We verified the performance of the model on the general pedestrian trajectory datasets. The experimental results show that our model has achieved state-of-the-art results in both long-term and short-term predictions for both high-density and low-density crowds.

## 2. Related Work

### 2.1. Pedestrian Trajectory Prediction

Pedestrian trajectory prediction has become a focal task in recent years, and corresponding solutions have been springing up. Comprehensively modelling the interactions between pedestrians is a crucial point to obtain better prediction results.

The article "MDST-DGCN: A Multilevel Dynamic Spatiotemporal Directed Graph Convolutional Network for Pedestrian Trajectory Prediction" was published in 2022. Journal: Comput Intell Neurosci.

Traditionally, researchers created hand-crafted functions [3, 6–10] to predict trajectories, but hand-crafted functions are limited, so they are unable to model all types of social interactions. Recently, deep learning-based methods have become popular because they can learn to model various interactions from data.

Some researchers designed their methods based on pooling mechanisms [11–14] to capture dependencies between pedestrians. The S-LSTM [11] introduces a “social” pooling layer which allows the LSTMs of spatially proximal sequences to share their hidden states with each other. Group-LSTM [12] adjusts the pooling layer by dropping the information of pedestrians who are moving coherently with the target pedestrian. MX-LSTM [13] has a pooling layer, which exploits the Vislet information. The above three pooling methods only consider the pedestrians in the local area and fuse their features averagely, while SGAN introduces a pooling module considering all pedestrians in a computationally efficient way and adaptively select their features with a max-pooling operation.

While most pooling-based methods treat pedestrians equally, attention-based methods [1, 15–20] assign different weights to interactive pedestrians. Most of these methods [1, 11–14, 16–20] assign an LSTM for each pedestrian, and the pooling mechanisms or the attention mechanisms usually work on the hidden states of pedestrians' LSTMs to adaptively fuse other pedestrians' motion features with the target pedestrian. More recently, STAR [28] captures complex spatiotemporal interactions by interleaving between spatial and temporal transformers [29].

As the graph structure is naturally suitable for directly describing the interactions between pedestrians, graph convolutional neural networks are introduced to this task. Social-BiGAT [21] replaced the pooling mechanisms with the graph attention network, which also works on the hidden states of LSTMs. In other words, Social-BiGAT did not model the whole duration of the crowds' interactions as a spatiotemporal graph but only used the graph attention network to capture the spatial social interactions. Social-STGCNN [23] and STGAT [22] both constructed spatiotemporal graphs to model social interactions. However, the graph of Social-STGCNN is a complete undirected graph. It does not conform to the asymmetry of pedestrian interactions. Zhang et al. [24] built a directed graph by inserting edges from all people inside the view area. However, all of these graphs model all the social interactions at only one level. Instead, we build a multilevel dynamic spatiotemporal directed graph to overcome their limitations.

The article "MDST-DGCN: A Multilevel Dynamic Spatiotemporal Directed Graph Convolutional Network for Pedestrian Trajectory Prediction" was published in 2022. Journal: Comput Intell Neurosci.

### 2.2. Graph Convolutional Neural Network

Graph convolutional neural network is an emerging topic in deep learning research, and it provides a practical approach to process graph data with nongrid structures. We can divide graph convolutional neural networks into spectral approaches [30–32] and spatial approaches [26, 33, 34]. Spectral approaches work with a spectral representation of the graphs, while spatial approaches define convolutions directly on the graph, operating on groups of spatially close neighbours. Spectral approaches' learned filters depend on the Laplacian eigenbasis, which depends on the graph structure. Thus, a model trained on a specific structure cannot be directly applied to a graph with a different structure. However, the graph used to model pedestrians' social interactions changes with time. Thus, spectral approaches are not suitable for pedestrian trajectory prediction. And, our approach belongs to the spatial approaches.

In fact, our approach follows the methodology of GraphSAGE [26]. However, our graph is a multilevel dynamic spatiotemporal directed graph, while GraphSAGE can only process a fixed spatial graph without multiple levels. ST-GCN [34] built a dynamic spatiotemporal graph to automatically learn both the spatial and temporal patterns of human actions to recognize skeleton-based actions. Social-STGCNN [23], which is a variant of ST-GCN that builds a single-level undirected graph to model all the social interactions, has achieved excellent results in pedestrian trajectory prediction.

## 3. Methods

### 3.1. Problem Definition

Given the historical trajectories of all pedestrians in the scenario, the task of trajectory prediction is to predict their future trajectories simultaneously. The notations *p*1, *p*_2_,…, *p*_*N*_ represent *N* pedestrians in the scenario. The position of a specific pedestrian *p*_*i*_(*i* ∈ [1, *N*]) at any historical time step *t*(*t* ∈ [1, *T*_obs_]) is defined as *X*_*i*_^*t*^=(*x*_*i*_^*t*^, *y*_*i*_^*t*^). Our goal is to predict the positions of pedestrians at any future time step *t*{*tɛ*[*T*_obs_+1+*T*_obs_+*T*_pred_]}, and for a specific pedestrian *p*_*i*_, the predicted position is denoted as ${\hat{Y}}_{i}^{t}=\left({\hat{x}}_{i}^{t},{\hat{y}}_{i}^{t}\right)$, while the ground truth is defined as *Y*_*i*_^*t*^=(*x*_*i*_^*t*^, *y*_*i*_^*t*^). The first-order difference trajectory of a pedestrian *p*_*i*_ is defined as {Δ*X*_*i*_^*t*^*|t* ∈ [1, *T*_obs_+*T*_pred_]}, where Δ*X*_*i*_^*t*^=*X*_*i*_^*t*^ − *X*_*i*_^*t*−1^.

The article "MDST-DGCN: A Multilevel Dynamic Spatiotemporal Directed Graph Convolutional Network for Pedestrian Trajectory Prediction" was published in 2022. Journal: Comput Intell Neurosci.

### 3.2. Overall Model

As shown in Figure 2(b), MDST-DGCN consists of three parts: a motion encoder, a multilevel dynamic spatiotemporal directed graph encoder (MDST-DGEN), and a motion decoder. The motion encoder is used to capture the pedestrian-specific motion features, and the MDST-DGEN is used to capture the social interaction features. We construct a multilevel dynamic spatiotemporal digraph processed by the MDST-DGEN to model the social interactions between pedestrians. After the motion features and social interaction features are extracted, they are fed into the motion decoder to predict future trajectories.

### 3.3. Graph Construction

We construct a multilevel dynamic spatiotemporal directed graph to model the multilevel social interactions between pedestrians. The nodes of the graph are the pedestrians in the scenario. Given the hyperparameter level distance list {*d*_1_, *d*_2_,…, *d*_*K*_}, we construct a graph with *K* levels. At each time step, if the distance from node *v*_*j*_ to node *v*_*i*_ is more than *d*_*k*−1_ and less than *d*_*k*_, a spatial edge from *v*_*j*_ to *v*_*i*_ will exist in the *k*_*th*_(*k* ∈ [1, *K*]) level. Specifically, in the 1_*st*_ level, a spatial edge exists when the distance is less than *d*_1_. For each node at all levels, we add a loop spatial edge. Figure 2(a) shows how to build a two-level spatial graph with the level distance list {*d*_1_, +*∞*} at a certain time step. In addition to spatial edges, there are temporal edges, which connect the same pedestrians in consecutive frames. If there is only one level and *d*_1_=+*∞*, the graph will degrade into a complete graph, which is of the same structure as STGAT. At the time step *t*, the attribute of node *v*_*i*_^*t*^ is the position *X*_*i*_^*t*^ of pedestrian *p*_*i*_.

### 3.4. Motion Encoder

The motion encoder is used to extract pedestrian-specific motion features. The input is the first-order difference trajectory {Δ*X*_*i*_^*t*^*|t* ∈ [1, *T*_obs_]}. The motion encoder is composed of a linear layer and an LSTM. The linear layer transforms the Δ*X*_*i*_^*t*^ into a higher dimension vector. Then, it is fed into the LSTM to get a motion feature vector. For each pedestrian *p*_*i*_, the process can be formulated as

(1) $$\begin{array}{c} h_{\text{mo}}^{t}\left(i\right)={\text{LSTM}}_{\text{mo}}\left(h_{\text{mo}}^{t-1}\left(i\right),{\text{Linear}}_{\text{en}}\left(\Delta X_{i}^{t};W_{\text{en}}\right);W_{\text{mo}}\right). \end{array}$$

Here, *W*_en_ denotes the trainable weights of the linear layer, *W*_mo_ is the trainable weights of the LSTM (LSTM_mo_), and the hidden states of LSTM_mo_ at the previous time step and the current time step of pedestrian *p*_*i*_ are denoted as *h*_mo_^*t*−1^(*i*) and *h*_mo_^*t*^(*i*), respectively. At last, the motion encoder obtains each pedestrian's motion feature vector *h*_mo_^*T*_obs_^(*i*), which is marked as *h*_mo_(*i*) in the following sections.

The article "MDST-DGCN: A Multilevel Dynamic Spatiotemporal Directed Graph Convolutional Network for Pedestrian Trajectory Prediction" was published in 2022. Journal: Comput Intell Neurosci.

### 3.5. MDST-DGEN

MDST-DGEN is a crucial component of our model. It processes the multilevel dynamic spatiotemporal directed social graph to obtain the social interaction features. If the graph is of *K* levels, MDST-DGEN will have *K* DGCN-LSTMs to process each level of it and an MSFM to fuse the features extracted from each level. In our implementation, *K* DGCN-LSTMs share the weights, so increasing the number of levels does not increase the parameters of the model.

### 3.6. DGCN-LSTM

After building the multilevel graph, each level of the graph is fed into a DGCN-LSTM. A DGCN-LSTM consists of a node aggregator architecture to process the spatial edges and an LSTM to process the temporal edges. We follow the design of GraphSAGE [26], which processes graphs by sampling and aggregating. Our node aggregator architecture generates embedding by sampling, aligning, and aggregating features from a node's spatial neighbourhood at each level.

#### 3.6.1. Sampling

Due to the different numbers of pedestrians in the scene, to process all nodes of different graphs in parallel, we expand the number of neighbours to a fixed number *m* by uniformly sampling a certain number of neighbours. Here, if there is an edge from node *v*_*j*_ to node *v*_*i*_, *v*_*j*_ will be the neighbour of *v*_*i*_. We denote the *m* neighbours of any node *v* as the neighbourhood set *𝒩*(*v*).

#### 3.6.2. Aligning

For the node *v*_*i*_, its attribute is the pedestrian's position *X*_*i*_^*t*^ and the attributes of its neighbourhood set can be denoted as {*X*_*j*_^*t*^*|*∀ *v*_*j*_ ∈ *𝒩*(*v*_*i*_)}. Social interaction is location independent, so we design an aligning operation to make the node aggregator architecture more generalizable. After aligning is done, the aligned attributes of any node *v*_*i*_'s neighbourhood set can be denoted as {*X*_*j*_^*t*^ − *X*_*i*_^*t*^*|*∀ *v*_*j*_ ∈ *𝒩*(*v*_*i*_)}. The intuitive understanding of the alignment operation is that we change the origin of coordinates to the position of node *v*_*i*_.

#### 3.6.3. Aggregating

After the aligning, we aggregate the aligned attributes of *v*_*i*_'s neighborhood set to obtain the new feature embedding of *v*_*i*_. It can be formulated as follows:

(2) $$\begin{array}{c} V_{i}^{t}=MAX\left(\left\{f\left(X_{j}^{t}-X_{i}^{t}\right)|\forall v_{j}\in N\left(v_{i}\right)\right\}\right), \end{array}$$

where MAX is the max operator that take the elementwise max of the transformed attribute vectors {*f*(*X*_*j*_^*t*^ − *X*_*i*_^*t*^)*|*∀ *v*_*j*_ ∈ *𝒩*(*v*_*i*_)} and *f* is the trainable linear mapping to convert a low-dimension vector to high dimension. We implement the max operator by using a max-pooling layer. Through the orderly use of sampling, aligning, and aggregating, our model can meet the requirement of a directed graph that the relation between two nodes in the directed graph is asymmetric.

The article "MDST-DGCN: A Multilevel Dynamic Spatiotemporal Directed Graph Convolutional Network for Pedestrian Trajectory Prediction" was published in 2022. Journal: Comput Intell Neurosci.

After the spatial edges are processed, an LSTM is used to process the temporal edges as follows:

(3) $$\begin{array}{c} h_{g}^{t}\left(i\right)={\text{LSTM}}_{g}\left(h_{g}^{t-1}\left(i\right),V_{i}^{t};W_{g}\right), \end{array}$$

where *W*_*g*_ is the trainable weights of the LSTM (LSTM_*g*_) and the hidden states of LSTM_*g*_ at previous time step and current time step are correspondingly denoted as *h*_*g*_^*t*−1^(*i*) and *h*_*g*_^*t*^(*i*). At last, the DGCN-LSTM obtains each pedestrian's social interaction feature vector *h*_*g*_^*T*_obs_^(*i*) at a certain level, and in the following sections, we denote *h*_*g*_^*T*_obs_^(*i*) of the *k*_*th*_ level as *H*_*g*_^*k*^(*i*).

### 3.7. MSFM

There are *K* levels in our graph, so there are *K* DGCN-LSTMs and the node *v*_*i*_'s social interaction feature vectors obtained by them can be denoted as {*H*_*g*_^1^(*i*), *H*_*g*_^2^(*i*),…, *H*_*g*_^*K*^(*i*)}. We use an MSFM to fuse all levels' social interaction feature vectors of node *v*_*i*_. The MSFM computes the weighted sum of {*H*_*g*_^1^(*i*), *H*_*g*_^2^(*i*),…, *H*_*g*_^*K*^(*i*)}. The formulations are as follows:

(4) $$\begin{array}{c} \alpha_{i}^{k}=\frac{\exp\left(h_{\text{mo}}{\left(i\right)}^{T}H_{g}^{k}\left(i\right)\right)}{\sum_{j\in \left[1,K\right]}\exp\left(h_{\text{mo}}{\left(i\right)}^{T}H_{g}^{j}\left(i\right)\right)},\\ H_{g}\left(i\right)=\sum_{k\in \left[1,K\right]}\alpha_{i}^{k}H_{g}^{k}\left(i\right). \end{array}$$

Here, *h*_mo_(*i*) is the motion feature vector of pedestrian *p*_*i*_, ·^*T*^ represents transposition, *H*_*g*_^*k*^(*i*) is the corresponding social interaction feature vector at level *k*, the fusion weight *α*_*i*_^*k*^ is a scalar, and *H*_*g*_(*i*) is the final fused social interaction feature vector.

### 3.8. Motion Decoder

The motion decoder is used to predict future trajectories based on the motion features and the fused social interaction features. There are two types of motion decoders: motion decoders without noise and motion decoders with noise. The former makes the whole model a deterministic one, and the latter makes it a stochastic one. For the deterministic type, we only concatenate *H*_*g*_(*i*) and *h*_mo_(*i*) as the initial hidden state of an LSTM and we train the model with L1 loss. For the stochastic type, we concatenate*H*_*g*_(*i*), *h*_mo_(*i*), and a noise vector *z* sampled from a standard Gaussian distribution to work as the initial hidden state of an LSTM. The formulation which shows how to get the initial hidden state of the stochastic motion decoder is as follows:

(5) $$\begin{array}{c} h_{\text{de}}\left(i\right)={\text{Linear}}_{h}\left(\text{concat}\left(H_{g}\left(i\right),h_{\text{mo}}\left(i\right),z\right);W_{h}\right). \end{array}$$

Moreover, we train the whole model with the variety loss proposed by SGAN [14] to encourage it to produce diverse samples. At the first prediction time step *T*_obs_+1, the decoder gets Δ*X*_*i*_^*T*_obs_^ as the initial input and predicts the next position offset $\Delta {\hat{X}}_{i}^{T_{\text{obs}}+1}$. The predicted position offset is marked as $\left\{\Delta {\hat{X}}_{i}^{t}|t\in \left[T_{\text{obs}}+1,T_{\text{obs}}+T_{\text{pred}}\right]\right\}$. The formulations which show how the stochastic motion decoder works are as follows:

(6) $$\begin{array}{c} h_{\text{de}}^{t}\left(i\right)={\text{LSTM}}_{\text{de}}\left(h_{\text{de}}^{t-1}\left(i\right),{\text{Linear}}_{\text{de}}\left(\Delta {\hat{X}}_{i}^{t};L_{\text{de}}\right);W_{\text{de}}\right),\\ \Delta {\hat{X}}_{i}^{t+1}={\text{Linear}}_{\text{pred}}\left(h_{\text{de}}^{t}\left(i\right);W_{\text{pred}}\right),\\ {\hat{Y}}_{i}^{t+1}={\hat{Y}}_{i}^{t}+\Delta {\hat{X}}_{i}^{t+1}, \end{array}$$

where *L*_de_ and *W*_pred_ are the trainable weights of the corresponding linear layers, concat means concatenating operation, and *W*_de_ denotes the trainable weights of the LSTM (LSTM_de_).

The article "MDST-DGCN: A Multilevel Dynamic Spatiotemporal Directed Graph Convolutional Network for Pedestrian Trajectory Prediction" was published in 2022. Journal: Comput Intell Neurosci.

## 4. Experiments

### 4.1. Datasets, Baseline Methods, and Metrics

#### 4.1.1. Datasets

We evaluate our method on three commonly used datasets, ETH [35], UCY [36], and a high-density pedestrian dataset, pedestrian walk path dataset [37], which is referred to as PEDWALK in the rest of the article. ETH and UCY contain 1536 pedestrians' real-world trajectories, while PEDWALK contains the manually labeled trajectories of 12684 pedestrians, and coordinates are provided in pixels. The image size of PEDWALK is 1920 × 1080 pixels. ETH and UCY consist of a total of five unique scenes: ETH, HOTEL (from ETH), ZARA1, ZARA2, and UNIV (from UCY). For ETH and UCY, we follow the leave-one-out evaluation methodology in SGAN [14], training on 4 scenes and testing on the remaining one. For PEDWALK, we use 70% of its total frames for training and leave the remaining 30% for evaluation. The interval of trajectory sequences of ETH and UCY is 0.4 seconds, while the interval of trajectory sequences of PEDWALK is 0.8 seconds. We take 8 ground truth positions as observation and predict the trajectories of the following 12 time steps. It means, for ETH and UCY, we observe for 3.2 seconds and predict the future at 4.8 seconds (short-term prediction), while for PEDWALK, we observe for 6.4 seconds and predict the future at 9.6 seconds (long-term prediction).

The article "MDST-DGCN: A Multilevel Dynamic Spatiotemporal Directed Graph Convolutional Network for Pedestrian Trajectory Prediction" was published in 2022. Journal: Comput Intell Neurosci.

#### 4.1.2. Baseline Methods

We compare MDST-DGCN of deterministic type (MDST-DGCN-D) with deterministic models, e.g., LSTM [27], S-LSTM [11], Social Attention [15], and CIDNN [19]. Furthermore, we compare MDST-DGCN of stochastic type (MDST-DGCN-S) with stochastic models, e.g., SGAN [14], SGAN-P [14], SoPhie [16], GAT [21], Social-BiGAT [21], STGAT [22], and Social-STGCNN [23].

#### 4.1.3. Metrics

There are two commonly used metrics: average displacement error (ADE) and final displacement error (FDE). ADE is the average L2 distance between ground truth and the predicted trajectory over all the predicted time steps, and FDE is the distance between the predicted final position and the actual final position at the end of the prediction period *T*_obs_+*T*_pred_. For stochastic models, similar to prior work [14, 22], 20 samples are generated and the closest sample to the ground truth is selected to compute ADE and FDE. After checking the codes of SGAN, STGAT, and Social-STGCNN, we find there are two different ways to select the closest sample: selecting the closest trajectory of each pedestrian in a sample used by Social-STGCNN [23] and selecting the closest sample used by SGAN [14] and STGAT [22]. A sample includes all pedestrians' trajectories in the scenario for a total duration of (*T*_obs_+*T*_pred_) time steps. Following the tradition of SGAN and STGAT, we select the closest sample to compute the ADE and FDE of MDST-DGCN-S.

### 4.2. Model Configuration and Training Details

For the motion encoder, the output dimension of the linear layer is 32 and the hidden state dimension of LSTM_mo_ is 64. For the MDST-DGEN, the output dimension of *f* and LSTM_*g*_ is 64. We implement *f* with a convolution layer. To process nodes in different scenarios in parallel, the fixed neighbour number *m* needs to be larger than the maximum number of pedestrians in a sample. The most crowded scene in PEDWALK contains 133 pedestrians, and in ETH and UCY, there are 57 pedestrians in the most crowded scene. So we set it 135 for PEDWALK and 60 for ETH and UCY. For the motion decoder, the output dimension of Linear_*h*_ is 32, the hidden state dimension of LSTM_de_ is 64, and the output dimension of Linear_pred_ is 2. For the MDST-DGCN-S, the dimension of the noise vector *z* is half of the hidden state dimension.

Our implementation is based on the PyTorch library. The model is trained on one NVIDIA GeForce GTX 1080Ti graphics card for 200 epochs. To calculate the variety loss with less GPU memory usage, we generate only 5 possible output predictions for each scene. In training, a batch size of 32 was used; we use the Adam optimizer with a learning rate of 0.0001. {1,5, +*∞*} is the default-level distance list for ETH and UNIV, and {150, +*∞*} is the default-level distance list for PEDWALK.

The article "MDST-DGCN: A Multilevel Dynamic Spatiotemporal Directed Graph Convolutional Network for Pedestrian Trajectory Prediction" was published in 2022. Journal: Comput Intell Neurosci.

### 4.3. Quantitative Evaluation

To validate the proposed MDST-DGCN, we present the prediction performance for both short-term trajectory prediction on ETH and UCY and long-term trajectory prediction on PEDWALK, and we present the prediction performance for various pedestrian densities. We elaborate on an ablation study to validate the effects of our multilevel graph and the aligning operation.

#### 4.3.1. MDST-DGCN-D

As Table 1 shows, MDST-DGCN-D outperforms all deterministic methods and some stochastic methods on ETH and UCY. And, as Table 2 shows, MDST-DGCN-D even outperforms stochastic methods including STGAT. It shows that our model has good performance in capturing interaction features, and we think there are three reasons. First, PEDWALK has many more pedestrians in a scene than ETH and UCY, and then it has more interaction types and more frequent interaction activities in a sample. Second, high-density limits the randomness of pedestrian movement. Third, the prediction horizon on PEDWALK is 9.6 s, while it is 4.8 s on ETH and UCY. When the prediction horizon is short, lots of decisions in movement occur in the observation period and continue to the prediction stage, so lots of useful cues exist in pedestrians' motion features and it is not necessary to infer from interactive information. High density and long-term predictions enhance the impact of interactions on trajectory prediction, and high density reduces the effect of multimodality.

#### 4.3.2. MDST-DGCN-S

As Tables 1 and 2 show, when the best sample of 20 predictions is selected to calculate ADE and FDE, MDST-DGCN-S outperforms all methods on PEDWALK and achieves comparable ADE and FDE with STGAT. The reasons why MDST-DGCN-S is not better than STGAT on ETH and UCY are the same as the reasons stated in (1). When the best trajectory of 20 predictions is selected, MDST-DGCN-S outperforms Social-STGCNN in ADE, but Social-STGCNN gets better FDEs in several subdatasets. It is mainly because there are accumulated errors when LSTM is used in our model.

#### 4.3.3. Various Pedestrian Densities

Table 2 presents the results on the PEDWALK for various pedestrian densities. We use samples with the specified densities to make the comparison. With the increase in density, the performance of each method decreases. Both MDST-DGCN-D and MDST-DGCN-S outperform other methods for various pedestrian densities. When the density is low, such as 10 ≤ *d* ≤ 30, the performance gap between SGAN and other methods is much smaller, which means when crowds are sparse, the effects of interactions are smaller and models get fewer useful cues to infer pedestrians' future movements, but the multimodality will work better. This phenomenon also confirms our previous reasoning in (1).

The article "MDST-DGCN: A Multilevel Dynamic Spatiotemporal Directed Graph Convolutional Network for Pedestrian Trajectory Prediction" was published in 2022. Journal: Comput Intell Neurosci.

#### 4.3.4. Different Level Distance Lists

Table 3 presents the ADEs and FDEs of MDST-DGCN-D with different level distance lists. The level distance list {+*∞*} means that MDST-DGCN-D models all social interactions at the same level, which is similar to STGAT and Social-STGCNN. Details about the level distance list are presented in Section 3. C. As shown in Table 3, modelling social interactions by a multilevel graph promotes the performance. On UNIV, the level distance list {1, +*∞*} helps MDST-DGCN-D to get the highest improvement. It is mainly because UNIV has a higher pedestrian density than the other four subdatasets, and more people will walk within one meter, the social comfort distance.

#### 4.3.5. Effects of Aligning Operation

As shown in Table 3, the aligning operation advances the performance on ETH, HOTEL, and UNIV, but it reduces the performance on ZARA1 and ZARA2. Because ZARA1 and ZARA2 are collected in the same place and have the same coordinate system, when they are used separately as a test set, the model without aligning will overfit on the coordinates.

### 4.4. Qualitative Evaluation

We compare the predicted trajectories of MDST-DGCN-D and STGAT in Figure 3. Figure 3(a) shows that the target pedestrian is walking in the same direction with a nearby pedestrian A, and he will finally gather with a faraway pedestrian B, both of STGAT and MDST-DGCN-D.

We successfully predict the merging phenomenon. However, MDST-DGCN-D succeeds in predicting that the target pedestrian maintains his relative position with nearby pedestrian A, while STGAT does not. Thus, MDST-DGCN-D obtains more accurate predictions. As shown in Figure 3(b), two pedestrians in a group are changing their directions in advance to avoid collisions with the pedestrians standing in the distance. For the target pedestrian, MDST-DGCN-D assigns a weight of 0.72 to the social interaction feature of the third level, which helps avoid possible collisions with distant pedestrians. However, STGAT only successfully predicts group behaviour but fails to predict early collision avoidance behaviour. All predictions in Figure 3 indicate that a multilevel graph structure can model social interactions more accurately and comprehensively.

The article "MDST-DGCN: A Multilevel Dynamic Spatiotemporal Directed Graph Convolutional Network for Pedestrian Trajectory Prediction" was published in 2022. Journal: Comput Intell Neurosci.

We also visualize the trajectory distributions of MDST-DGCN-S and STGAT in Figure 4. As shown in Figure 4, in all three samples of pedestrian avoidance, pedestrian following, and pedestrian walking in group, our model outperforms STGAT.

We count the distribution of fusion weight (*α*) on PEDWALK, which shows that the social interaction features of the first level and second level are of different importance in a sample. The distribution of fusion weight (*α*) is shown in Figure 5.

## 5. Conclusions

In this article, we propose a multilevel dynamic spatiotemporal directed graph representation to model the interactions between pedestrians and introduce MDST-DGCN to process the multilevel graph. Experimental results indicate that our multilevel graph structure can model social interactions more accurately and comprehensively and show that MDST-DGCN outperforms most of the state-of-the-art methods.

## Figures and Tables

**Figure 1:** The influences of pedestrians in the nearby area and the faraway area on the target pedestrian are more suitable to be modeled separately at different levels.

**Figure 2:** (a) Illustration of how to build a two-level spatial graph with the level distance list {*d*_1_, +*∞*} at a certain time step. Level 1 shows the relation between pedestrians within the distance of *d*_1_, and Level 2 shows it beyond the distance of *d*_1_. The left graphs show the edges from others to a specific pedestrian at different levels, and the right ones show all edges in the graphs of different levels. (b) The architecture of MDST-DGCN.

**Figure 3:** Qualitative comparison between MDST-DGCN-D and STGAT. For better visualization, only a few trajectories are drawn and we draw the area of each level at the last historical time step.

**Figure 4:** Trajectory distribution visualization for MDST-DGCN-S and STGAT. For better visualization, only a few trajectories are drawn.

**Figure 5:** The distribution of fusion weight (*α*). Alpha of h is the fusion weight of the hidden state, and alpha of c is the fusion weight of the cell state.

**Table 1:** We compare deterministic baseline models with MDST-DGCN of deterministic type (MDST-DGCN-D) and stochastic baseline models with MDST-DGCN of stochastic type (MDST-DGCN-S) on ETH and UCY.

Method	ETH	HOTEL	UNIV	ZARA1	ZARA2	AVG

LSTM [14, 27]	1.09/2.41	0.86/1.91	0.61/1.31	0.41/0.88	0.52/1.11	0.70/1.52
S-LSTM [11, 14]	1.09/2.35	0.79/1.76	0.67/1.40	0.47/1.00	0.56/1.17	0.72/1.54
Social Attention [15, 22]	1.39/2.39	2.51/2.91	1.25/2.54	1.01/2.17	0.88/1.75	1.41/2.35
CIDNN [19, 22]	1.25/2.32	1.31/2.36	0.90/1.86	0.50/1.04	0.51/1.07	0.89/1.73
MDST-DGCN-D	**0.86/1.75**	**0.44/0.90**	**0.55/1.16**	**0.40/0.86**	**0.32/0.68**	**0.51/1.07**

SoPhie^*∗*1^ [16]	0.70/1.43	0.76/1.67	0.54/1.24	0.30/0.63	0.38/0.78	0.54/1.15
GAT^*∗*1^ [21]	0.68/1.29	0.68/1.40	0.57/1.29	0.29/0.60	0.37/0.75	0.52/1.07
Social-BiGAT^*∗*1^ [21]	0.69/1.29	0.49/1.01	0.55/1.32	0.30/0.62	0.36/0.75	0.48/1.00
SGAN^*∗*2^ [14]	0.81/1.52	0.72/1.61	0.60/1.26	0.34/0.69	0.42/0.84	0.58/1.18
SGAN-p^*∗*2^ [14]	0.87/1.62	0.67/1.37	0.76/1.52	0.35/0.68	0.42/0.84	0.61/1.21
STGAT^*∗*2^ [22]	**0.65/1.12**	0.35/0.66	0.52/**1.10**	0.34/**0.69**	0.29/0.60	**0.43/0.83**
MDST-DGCN-S^*∗*2^	0.69/1.45	**0.34/0.58**	**0.51**/1.11	**0.33**/0.70	**0.28/0.59**	**0.43**/0.89

Social-STGCNN^*∗*3^ [23]	0.64/**1.11**	0.49/0.85	0.44/**0.79**	0.34/**0.53**	0.30/0.48	0.44/0.75
MDST-DGCN-S3	**0.56**/1.12	**0.27/0.50**	**0.38**/0.81	**0.27**/0.56	**0.22/0.46**	**0.34/0.69**

We predict future at 4.8 seconds (short-term prediction), given the previous 3.2 seconds. The errors reported are ADE or FDE in meters. Methods marked with *∗* draw 20 samples. The ADE and FDE of methods marked with superscript 2 are calculated by selecting the closest sample; the ADE and FDE of methods marked with superscript 3 are calculated by selecting the closest trajectory; and for the ADE and FDE of methods marked with superscript 1, we are not sure which type they belong to, because we cannot find their code. The values with the least error in the comparison model are bolded.

The article "MDST-DGCN: A Multilevel Dynamic Spatiotemporal Directed Graph Convolutional Network for Pedestrian Trajectory Prediction" was published in 2022. Journal: Comput Intell Neurosci.

**Table 2:** ADEs and FDEs of different methods for long-term trajectory prediction on the PEDWALK with various pedestrian densities.

Density (d)	10 ≤ d ≤ 30	30 ≤ d ≤ 50	50 ≤ d ≤ 70	70 ≤ d ≤ +∞	Overall

SGAN*∗*	35.57/70.39	44.02/87.08	43.30/85.84	47.34/93.24	44.02/86.96
SGAN-P*∗*	36.06/71.02	41.92/81.39	40.70/78.70	45.09/87.39	42.03/81.54
STGAT*∗*	33.20/60.21	38.06/68.25	38.33/69.18	41.97/75.98	39.02/70.47
MDST-DGCN-D	**32.62**/63.05	**36.38**/69.15	**35.61/67.17**	**40.80**/77.77	**37.31**/70.80
MDST-DGCN-S*∗*	**30.53/57.88**	**34.62/64.81**	**34.68/64.81**	**39.75/75.21**	**35.99/67.53**

The density (d) means the number of pedestrians in the scenario, and D1 ≤ d ≤ D2 means we select the samples in which the number of pedestrians is not less than D1 and not greater than D2. All methods predict 9.6 seconds, given the previous 6.4 seconds. Errors reported are ADE/FDE in pixels on the original size of 1920 × 1080. Methods marked with *∗* draw 20 samples and select the best sample. The values with the least error in the comparison model are bolded.

**Table 3:** Ablation study of MDST-DGCN-D with different level distance lists and with or without aligning operation for short-term prediction on ETH and UCY.

Level distance list	ETH	HOTEL	UNIV	ZARA1	ZARA2	AVG

{+∞}	0.870/1.792	0.490/1.011	0.626/1.273	0.407/0.867	0.333/0.703	0.545/1.129
{1, +∞}	0.862/1.772	0.465/0.989	**0.532/1.139**	0.402/0.862	0.324/0.687	0.517/1.090
{5, +∞}	**0.853**/1.757	0.453/0.931	0.624/1.269	0.400/0.852	0.322/0.684	0.530/1.100
{1, 5, +∞}*∗*	0.859/**1.749**	**0.437/0.900**	0.547/1.161	0.402/0.860	0.320/0.684	**0.513/1.071**
Without aligning	0.90/1.94	1.48/2.49	0.60/1.25	**0.37/0.79**	**0.30/0.65**	0.73/1.42

The level distance list {1, 5, +∞}*∗* is the default setting, and it is used for MDST-DGCN-D without aligning operation. The errors reported are ADE or FDE in meters. The values with the least error in the comparison model are bolded.

The article "MDST-DGCN: A Multilevel Dynamic Spatiotemporal Directed Graph Convolutional Network for Pedestrian Trajectory Prediction" was published in 2022. Journal: Comput Intell Neurosci.

## Data Availability

Previously reported ETH and UCY data were used to support this study and are available at https://doi.org/10.1109/ICCV.2009.5459260 and https://doi.org/10.1111/j.1467-8659.2007.01089.x. These prior studies are cited at relevant places within the text as references. Previously reported PEDWALK data were used to support this study and are available at https://doi.org/10.1109/CVPR.2015.7298971. The prior study is cited at relevant places within the text as references.

## References

[1] Ma Y., Zhu X., Zhang S., Yang R., Wang W., Manocha D. (2019). Trafficpredict: trajectory prediction for heterogeneous traffic-agents. *Proceedings of the AAAI Conference on Artificial Intelligence*.

[2] Bennewitz M., Burgard W., Cielniak G., Thrun S. (2005). Learning motion patterns of people for compliant robot motion. *The International Journal of Robotics Research*.

[3] Pradhan N., Burg T., Birchfield S. Robot crowd navigation using predictive position fields in the potential function framework.

[4] Chen Z., Song C., Yang Y. (2018). Robot navigation based on human trajectory prediction and multiple travel modes. *Applied Sciences*.

[5] Chinag C., Ding C. Robot navigation in dynamic environments using fuzzy logic and trajectory prediction table.

[6] Ma Y., Manocha D., Autorvo W. W. (2018). Local navigation with dynamic constraints in dense heterogeneous traffic. https://arxiv.org/abs/1804.02915.

[7] Mehran R., Oyama A., Shah M. Abnormal crowd behavior detection using social force model.

[8] Helbing D., Molnár P. (1995). Social force model for pedestrian dynamics. *Physical Review A*.

[9] Tian L., Collins C. (2004). An effective robot trajectory planning method using a genetic algorithm. *Mechatronics*.

[10] Richards A., How J. P. Aircraft trajectory planning with collision avoidance using mixed integer linear programming.

[11] Alahi A., Goel K., Ramanathan V., Robicquet A., Fei-Fei L., Savarese S. Social LSTM: human trajectory prediction in crowded spaces.

The article "MDST-DGCN: A Multilevel Dynamic Spatiotemporal Directed Graph Convolutional Network for Pedestrian Trajectory Prediction" was published in 2022. Journal: Comput Intell Neurosci.

[12] Bisagno N., Zhang B., Conci N. Group LSTM: group trajectory prediction in crowded scenarios.

[13] Hasan I., Setti F., Tsesmelis T., Del Bue A., Galasso F., Cristani M. MX-LSTM: mixing tracklets and vislets to jointly forecast trajectories and head poses.

[14] Gupta A., Johnson J., Fei-Fei L., Savarese S., Alahi A. Social GAN: socially acceptable trajectories with generative adversarial networks.

[15] Vemula A., Muelling K., Oh J. Social Attention: modeling attention in human crowds.

[16] Sadeghian A., Kosaraju V., Sadeghian A., Hirose N., Rezatofighi H., Savarese S. SoPhie: an attentive gan for predicting paths compliant to social and physical constraints.

[17] Liang J., Jiang L., Niebles J. C., Hauptmann A. G., FeiFei L. Peeking into the future: predicting future person activities and locations in videos.

[18] Zhang P., Ouyang W., Zhang P., Xue J., Zheng N. SR-LSTM: state refinement for lstm towards pedestrian trajectory prediction.

[19] Xu Y., Piao Z., Gao S. Encoding crowd interaction with deep neural network for pedestrian trajectory prediction.

[20] Amirian J., Hayet J., Pettr J. Social Ways: learning multi-modal distributions of pedestrian trajectories with GANs.

[21] Kosaraju V., Sadeghian A., Mart´ın-Mart´ın R., Reid I., Rezatofighi H., Savarese S. (2019). Social-BiGAT: multimodal trajectory forecasting using Bicycle-GAN and graph attention networks. *Advances in Neural Information Processing Systems*.

[22] Huang Y., Bi H., Li Z., Mao T., Wang Z. STGAT: modeling spatial-temporal interactions for human trajectory prediction.

[23] Mohamed A., Qian K., Elhoseiny M., Claudel C. Social-STGCNN: a social spatio-temporal graph convolutional neural network for human trajectory prediction.

[24] Zhang L., She Q., Guo P. (2019). Stochastic trajectory prediction with social graph network. https://arxiv.org/abs/1907.10233.

[25] Ivanovic B., Pavone M. The Trajectron: probabilistic multi-agent trajectory modeling with dynamic spatiotemporal graphs.

[26] Hamilton W., Ying R., Leskovec J. (2017). Inductive representation learning on large graphs. *Advances in Neural Information Processing Systems*.

[27] Hochreiter S., Schmidhuber J. (1997). Long short-term memory. *Neural Computation*.

[28] Yu C., Ma X., Ren J., Zhao H., Yi S. Spatio-temporal graph transformer networks for pedestrian trajectory prediction.

[29] Vaswani A., Shazeer N., Parmar N. Attention is all you need.

[30] Joan B., Wojciech Z., Arthur S., Yann L. (2013). Spectral networks and locally connected networks on graphs. https://arxiv.org/abs/1312.6203.

[31] Michael D., Xavier B., Pierre V. (2016). Convolutional neural networks on graphs with fast localized spectral filtering. *Advances in Neural Information Processing Systems*.

The article "MDST-DGCN: A Multilevel Dynamic Spatiotemporal Directed Graph Convolutional Network for Pedestrian Trajectory Prediction" was published in 2022. Journal: Comput Intell Neurosci.

[32] Kipf T., Welling M. Semi-supervised classification with graph convolutional networks.

[33] Velickovic P., Cucurull G., Casanova A., Romero A., Lio P., Bengio Y. Graph attention networks.

[34] Yan S., Xiong Y., Lin D. Spatial temporal graph convolutional networks for skeleton-based action recognition.

[35] Pellegrini S., Ess A., Schindler K., van Gool L. You’ll never walk alone: modeling social behavior for multi-target tracking.

[36] Alon L., Yiorgos C., Dani L. (2007). Crowds by example. *Computer Graphics Forum*.

[37] Yi S., Li H., Wang X. Understanding pedestrian behaviors from stationary crowd groups.

